# Therapeutic Value of Traditional Chinese Massage plus Moxibustion for Degenerative Knee Osteoarthritis

This article has been retracted.

**DOI:** 10.1155/2022/8305561

**Published:** 2022-06-30

**Authors:** Jianhui Yang, Jianping Zou, Qingfeng Zhang

**Affiliations:** Department of Pain, First Affiliated Hospital of Xian Jiaotong University, Xi'an 710061, China

## Abstract

**Objective:**

To evaluate the therapeutic value of traditional Chinese massage plus moxibustion for degenerative knee osteoarthritis (DKOA).

**Methods:**

From January 2019 to October 2021, 152 patients with DKOA were enrolled. All patients were randomly divided into the treatment group and the control group. The control group was treated with oral glucosamine hydrochloride capsules. The treatment group was treated with traditional Chinese massage and moxibustion on the basis of the control group. The duration of treatment in the two groups was 8 weeks. The effectiveness, visual analog scale (VAS) score, the hospital for special surgery (HSS) score, World Health Organization Quality of Life Scale (WHOQOL-BREF) score, serum high-sensitivity C-reactive protein (CRP), and interleukin-6 (IL-6) levels were compared between the two groups before and after treatment.

**Results:**

There were no significant differences in age, sex, and the duration of disease between the two groups (*P* > 0.05). The overall response rate in the treatment group was significantly higher than that of the control group after treatment (92.1% vs 78.9%; *P*=0.038); the VAS score of both two groups were significantly decreased, and the VAS score in the treatment group was significantly lower than that of the control group (3.5 ± 1.4 vs 4.8 ± 1.1; *P* < 0.001); the HSS score and WHOQOL-BREF score significantly improved in both groups, and the HSS score and WHOQOL-BREF score improved more in the treatment group than those of the control group (*P* < 0.05). The high-sensitivity CRP level significantly decreased in both groups, and the high-sensitivity CRP level in treatment group is lower than that of the control group (2.79 ± 1.65 vs 4.37 ± 1.54; *P* < 0.001); the IL-6 level was significantly decreased in the treatment group than in the control group (7.22 ± 3.41 vs 4.59 ± 2.98; *P* < 0.001).

**Conclusion:**

Traditional Chinese massage plus moxibustion is worthy of clinical application, which has a significant clinical effect on DKOA, reducing pain and improving knee joint function and quality of life.

## 1. Introduction

Degenerative osteoarthritis (DOA) is a common osteoarticular disease. Degenerative knee arthritis (DKOA) is the most common in DOA, mainly manifested as joint stiffness with limited mobility, persistent pain, or motor pain with numbness [1]. Patients with DKOA have mild initial symptoms, mainly joint stiffness with alleviation after activity, varying degrees of joint swelling and deformation, and limited mobility with significant pain in the later stage of the disease [2]. In general, any damaging factor affecting joint biomechanics causes or aggravates DKOA in addition to age and subsequently leads to clinical symptoms [3]. The knee joint is an important weighing joint of body. The occurrence of DKOA can seriously affect the walking ability and quality of life [4] and may be associated with a subsequent increase in the risk of falls and fractures [5]. There are many clinical treatments for DKOA, including conservative treatment such as oral glucosamine, local injection of sodium hyaluronate, and physical therapy. Nonsteroidal anti-inflammatory drugs and local blocking can be used to relieve local pain and improve joint activity when the pain is obvious [6]. However, the disadvantage of conservative treatment is slow and fair effect, long course, and high cost. It is urgent to find an effective treatment for DKOA. Traditional Chinese massage is a standardized manual therapy which is performed by well-trained TCM medical staff with high safety and is widely accepted by patients [7]. Traditional Chinese medicine (TCM) is the system with the longest history and is gaining popularity in other countries too [8]. Previous studies show that traditional Chinese medicine have been used in different ethnics and races [9, 10]. Moxibustion therapy, an important way of TCM treatment, is mainly through the heat of moxibustion to give warm stimulation and activate meridian acupoints, so as to improve the clinical symptoms of patients [11]. There are still few studies on traditional Chinese massage combined with moxibustion in the treatment of DKOA. In this study, we observed the effectiveness, visual analog scale (VAS) score, the hospital for special surgery (HSS) score, World Health Organization Quality of Life Scale (WHOQOL-BREF) score, serum high-sensitivity C-reactive protein (CRP), and interleukin-6 (IL-6) level after treatment to evaluate the value of traditional Chinese massage plus moxibustion in the treatment of DKOA.

## 2. Patients and Methods

### 2.1. Patients

From January 2019 to October 2021, 152 patients with DKOA were enrolled. Inclusion criteria were as follows: (1) ≥18 years old; (2) combined with the clinical symptoms, signs, and X-ray and other typical imaging findings, in line with the diagnostic criteria of degenerative gonarthritis; (3) without surgical treatment, understanding the treatment plan, and agreeing to conservative treatment.

Exclusion criteria were as follows: (1) infectious arthritis, rheumatoid arthritis, or traumatic arthritis; (2) serious organ dysfunction; (3) blood system diseases or malignant tumors; (4) mental disorders or cannot cooperate to complete the treatment; (5) other situation which could affect the levels of high-sensitivity CRP and IL-6. This study was approved by the Ethics Committee of First Affiliated Hospital of Xian Jiaotong University. All patients signed informed consent forms.

### 2.2. Grouping and Treatment

The patients were randomly divided into the treatment group and control group. The control group was treated with oral glucosamine hydrochloride capsules, 0.75 g twice daily (Hong Kong Aussie Pharmaceutical Factory) for 8 weeks. On the basis of the control group, the treatment group was treated with traditional Chinese massage plus moxibustion three times a week for 8 weeks.

The treatment plan of traditional Chinese massage plus moxibustion was as follows: assist the patient to lie in the supine position, place the bolster under the knee, and use a rolling massage and a finger-Zen pushing method to treat the knee joint and its surroundings; the massage site starts from the distal knee joint, and the massage time lasts for 5 minutes. Then, acupoints such as Zusanli, Yanglingquan, Liangqiu, and Xuehai were taken for point pressing, each lasting 2 minutes. At the end of the massage, a moxibustion box was placed on the affected knee, and moxa sticks were placed according to acupoints such as Eryanglingquan, Yinlingquan, Xuehai, Liangqiu and internal and external knee eyes, Zusanli and Chengshan, to ignite moxa stick fumigation moxibustion for about 30 minutes.

### 2.3. Outcome Measures

Efficacy was assessed using the following outcome measures. (1) Outcomes: markedly effective is defined as the basic disappearance of symptoms, basically normal joint function, and the ability to complete daily life and work; effective is defined as significant relief of symptoms, significant improvement of joint function, and improvement in the ability to participate in activities or work; and ineffective is defined as no improvement in symptoms and signs. Overall response rate = (markedly effective + effective)/total number of cases × 100%. (2) VAS score: the degree of pain was assessed using the visual analog scale (VAS) score, ranging from 0 to 10 [12]. (3) HSS score: the Hospital for Special Surgery (HSS) score was used to evaluate the knee joint function [13]. The scale included seven items: pain degree, joint function, joint range of motion, etc. (4) WHOQOL-BREF score: World Health Organization Quality of Life Scale (WHOQOL-BREF) was used [14] to evaluate patient's quality of life. (5) High-sensitivity CRP and IL-6: 10 mL fasting venous blood was drawn before and after treatment and was placed for 10min and centrifuged to obtain the upper serum, and high-sensitivity CRP and IL-6 levels were measured by ELISA.

### 2.4. Statistical Analysis

Statistical analysis was performed by IBM SPSS 21.0. Categorical variables were expressed as *n* (%), and differences were compared using the chi-square test. Continuous variables were expressed as mean ± SD, and *t*-test was used to compare differences. The *t*-test was used to compare the differences in VSS score, HSS score, WHOQOL-BREF score, high-sensitivity CRP level, and IL-6 level before and after treatment. *P* < 0.05 was considered to be statistically significant.

## 3. Results

### 3.1. Clinical Characteristics

As shown in Table 1, a total of 152 patients with DKOA were included. There are 76 patients in the treatment group (age: 64.6 ± 9.7 years, male: 46, 60.5%), and the duration of disease was 2.49 ± 0.82 years. There are 76 patients in the treatment group (age: 63.1 ± 8.7 years, male: 48, 63.2%), and the duration of disease was 2.31 ± 0.77 years. There were no significant differences in age, sex, and duration of disease between the two groups (*P* > 0.05).

### 3.2. Treatment Outcomes

As shown in Table 2 and Figure 1, the number of markedly effective, effective, and ineffective patients in the treatment group was 44, 26, and 6, respectively. The number of markedly effective, effective, and ineffective patients in the control group was 32, 28, and 16, respectively. The overall response rate in the treatment group was significantly higher than that in the control group (92.1 vs 78.9%, *P*=0.038).

### 3.3. VAS Score

As shown in Table 3, the VAS score of the treatment group showed no significant difference comparred to the control group (7.6 ± 1.3 vs 7.8 ± 1.0; *P*=0.238) before treatment. The VAS score was significantly decreased in both groups after treatment, and the VAS score in the treatment group was significantly lower than that in the control group (3.5 ± 1.4 vs 4.8 ± 1.1, *P* < 0.001).

### 3.4. HSS Score and WHOQOL-BREF Score

As shown in Table 4, there was no significant difference in the HSS score (41.6 ± 6.7 vs 42.4 ± 7.1, *P*=0.496) and WHOQOL-BREF score (53.8 ± 7.8 vs 55.3 ± 8.4, *P*=0.246) between the two groups before treatment. The HSS score was significantly increased after treatment in both groups, and the HSS score in the treatment group was significantly higher than that in the control group (80.2 ± 6.8 vs 72.1 ± 7.3, *P* < 0.001). The WHOQOL-BREF score was significantly increased, and the WHOQOL-BREF score in the treatment group was increased more than that in the control group (65.6 ± 8.9 vs 74.0 ± 8.7, *P* < 0.001).

### 3.5. High-Sensitivity C-Reactive Protein (hs-CRP) and Interleukin-6 (IL-6) Levels

As shown in Table 5, there was no significant difference in the high-sensitivity CRP level (7.82 ± 2.20 vs 7.30 ± 1.43, *P*=0.088) and IL-6 (9.91 ± 3.43 vs 10.33 ± 3.36, *P*=0.446) in the treatment group compared to the control group. The high-sensitivity CRP level of both groups decreased significantly after treatment, and the high-sensitivity CRP level in the treatment group was significantly lower than that in the control group (2.79 ± 1.65 vs 4.37 ± 1.54; *P* < 0.001). The IL-6 levels significantly decreased in both groups after treatment, and the IL-6 levels in the treatment group was significantly lower than that in the control group (7.22 ± 3.41 vs 4.59 ± 2.98, *P* < 0.001).

## 4. Discussion

In this study, the patients with traditional Chinese massage plus moxibustion regimen could reduce pain symptoms, improve knee function and quality of life, and reduce the levels of inflammatory factors such as high-sensitivity CRP and IL-6, and it could effectively treat DKOA.

Previous studies suggest that the prevalence of DKOA is between 4.2% and 15.5%, which is associated with age and region [15]. It is estimated that the prevalence of symptomatic gonarthritis is 8.1% in the Chinese population, which is higher in women than men and in rural areas than towns. The prevalence of gonarthritis diagnosed by imaging may be 8.1% [4]. Therefore, DKOA is a heavy burden for both society and families. At present, the main mechanism of DKOA may be due to biomechanical factors caused by chondrocyte, extracellular matrix, and subchondral bone anabolic and catabolic imbalance. Age, obesity, occupation, ethnicity, endocrine hormones, and genetic factors are all thought to be associated with the pathogenesis of DKOA [16]. DKOA belongs to the category of “Bi Zheng” according to TCM, which is a disease caused due to evil qi such as wind, cold, dampness, and heat blocking meridians, affecting the movement of qi and blood, resulting in pain, numbness, or the presence of symptoms such as joint movement disorders in joints and muscles [17]. In this study, we improved the metabolism of tissues around the knee joint, reduced intra-articular pressure, and promoted the repair of intra-articular tissues through traditional Chinese massage [18]. Moxibustion can promote blood circulation, release bone and joint adhesions, and regulate joint tension and balance [19]. The combination of the two can effectively treat DKOA.

Notably, this study also found that traditional Chinese massage combined with moxibustion treatment could reduce the levels of inflammatory factors, including high-sensitivity CRP and IL-6. High-sensitivity CRP is a common inflammatory factor that is mainly produced by hepatocytes during the inflammatory response, and the production of high-sensitivity CRP is significantly correlated with the activity of the inflammatory response [20]. It has been suggested that patients with osteoarthritis have mildly elevated high-sensitivity CRP concentrations and the concentration of high-sensitivity CRP is significantly associated with pain and limb movement disorders [21]. IL-6 is also an important inflammatory factor, mainly produced by lymphocytes, and IL-6 and high-sensitivity CRP are involved in the activation of the inflammatory response and play an important role in the development of DKOA [2]. In this study, after treatment with traditional Chinese massage plus moxibustion, the high-sensitivity CRP and IL-6 levels of both groups decreased significantly and the levels in the treatment group were significantly lower than in the control group. We hypothesize that traditional Chinese massage combined with moxibustion may treat DKOA by reducing inflammatory activity and improving the mechanism of inflammatory response [19].

This study has the following limitations: small sample size, short study time, and collection of fewer variables.

In summary, the traditional Chinese massage plus moxibustion regimen can significantly improve the pain symptoms and quality of life of patients with DKOA, restore knee function, and reduce high-sensitivity CRP and IL-6 levels, which is worthy of clinical promotion. Future interventional trials with large samples are needed to further validate the effect of traditional Chinese massage plus moxibustion regimen in patients with DKOA.

## Figures and Tables

**Figure 1:** Treatment response rate.

**Table 1:** Clinical characteristics.

	Treatment group (*n* = 76)	Control group (*n* = 76)	*T*/*χ*^2^	*P* value
Age, years	64.6 ± 9.7	63.1 ± 8.7	1.042	0.299
Sex, *n* (%)			0.112	0.738
Male	46 (60.5)	48 (63.2)		
Female	30 (39.5)	28 (36.8)		
Disease duration, *y*	2.49 ± 0.82	2.31 ± 0.77	1.437	0.153

**Table 2:** Treatment response rate.

	Markedly effective	Effective	Invalid	Overall response rate, *b*%
Treatment group (*n* = 76)	44 (57.9)	26 (34.2)	6 (7.9)	92.1
Control group (*n* = 76)	32 (42.1)	28 (36.8)	16 (21.1)	78.9
Χ^2^	6.514			
*P* value	0.038			

**Table 3:** VAS scores.

	Before treatment	After treatment	*T*	*P* value
Treatment group (*n* = 76)	7.6 ± 1.3	3.5 ± 1.4	18.515	<0.001
Control group (*n* = 76)	7.8 ± 1.0	4.8 ± 1.1	17.593	<0.001
*T* value	−1.184	−6.452	—	—
*P* value	0.238	<0.001	—	—

**Table 4:** HSS score and WHOQOL-BREF score of patients.

	HSS score		WHOQOL-BREF score	
	Before treatment	After treatment	Before treatment	After treatment
Treatment group (*n* = 76)	41.6 ± 6.7	80.2 ± 6.8^*∗*^	53.8 ± 7.8	74.0 ± 8.7^*∗*^
Control group (*n* = 76)	42.4 ± 7.1	72.1 ± 7.3^*∗*^	55.3 ± 8.4	65.6 ± 8.9^*∗*^
*T* value	−0.683	7.088	−1.165	5.873
*P* value	0.496	<0.001	0.246	<0.001

^*∗*^ *P* < 0.001, compared with pretreatment in the same group.

**Table 5:** High-sensitivity C-reactive protein (hs-CRP) and interleukin-6 (IL-6) levels.

	Hs-CRP (mg/L)		IL-6 (pg/L)	
	Before treatment	After treatment	Before treatment	After treatment
Treatment group (*n* = 76)	7.82 ± 2.20	2.79 ± 1.65 ^*∗*^	9.91 ± 3.43	4.59 ± 2.98^*∗*^
Control group (*n* = 76)	7.30 ± 1.43	4.37 ± 1.54^*∗*^	10.33 ± 3.36	7.22 ± 3.41^*∗*^
*T* value	1.717	−6.079	−0.764	−5.067
*P* value	0.088	<0.001	0.446	<0.001

^*∗*^ *P* < 0.001, compared with pretreatment in the same group.

## Data Availability

The data used to support the findings of this study are available from the corresponding author upon request.
